The article "Structural insights into interactions between viral suppressor of RNA silencing protein p19 mutants and small RNAs" was published in 2019. Journal: FEBS Open Bio.

# Structural insights into interactions between viral suppressor of RNA silencing protein p19 mutants and small RNAs

**DOI:** 10.1002/2211-5463.12644

**Published:** 2019-05-17

**Authors:** Dana V. Foss, Nicole T. Schirle, Ian J. MacRae, John Paul Pezacki

**Affiliations:** ^1^ Department of Biochemistry, Microbiology and Immunology University of Ottawa Canada; ^2^ Department of Integrative Structural and Computational Biology The Scripps Research Institute La Jolla CA USA; ^3^ Department of Chemistry and Biomolecular Sciences University of Ottawa Canada

**Keywords:** engineering RNA binding proteins, p19 protein, protein:RNA interactions, X‐ray crystallography of protein:RNA complex

## Abstract

Viral suppressors of RNA silencing (VSRSs) are a diverse group of viral proteins that have evolved to disrupt eukaryotic RNA silencing pathways, thereby contributing to viral pathogenicity. The p19 protein is a VSRS that selectively binds to short interfering RNAs (siRNAs) over microRNAs (miRNAs). Mutational analysis has identified single amino acid substitutions that reverse this selectivity through new high‐affinity interactions with human miR‐122. Herein, we report crystal structures of complexed p19‐T111S (2.6 Å), p19‐T111H (2.3 Å) and wild‐type p19 protein (2.2 Å) from the Carnation Italian ringspot virus with small interfering RNA (siRNA) ligands. Structural comparisons reveal that these mutations do not lead to major changes in p19 architecture, but instead promote subtle rearrangement of residues and solvent molecules along the p19 midline. These observations suggest p19 uses many small interactions to distinguish siRNAs from miRNAs and perturbing these interactions can create p19 variants with novel RNA‐recognition properties.

**Database:**

Model data are deposited in the PDB database under the accession numbers 6BJG, 6BJH and 6BJV.

**Abbreviations**
AGO: Argonaute
CIRV: Carnation Italian ringspot virus
dsRNA: double‐stranded RNA
His8‐tag: octa‐histidine tag
miRNA: microRNA
nt: nucleotide
RISC: RNA‐induced silencing complex
RNAi: RNA interference
siRNA: short interfering RNA
ssRNA: single‐stranded RNA
TBSV: tomato bushy stunt virus
VSRS: viral suppressor of RNA silencing

## p19 viral suppressor of RNA silencing

The RNA silencing pathway plays a major role in viral defence in plants and invertebrates, where double‐stranded RNA molecules generated during viral replication are recognized by the Dicer enzyme, generating siRNAs. siRNA duplexes are bound by host Argonaute proteins, which unwind the duplex and use one strand as a guide to target and silence complementary sequences in the viral genome, via the RNA‐induced silencing complex (RISC). VSRSs are a diverse group of viral proteins that have evolved to disrupt eukaryotic RNA silencing pathways, thereby contributing to viral pathogenicity 1. Some VSRSs interfere directly with the silencing machinery of the host plant 2, 3, 4. Several VSRSs interact with dsRNA, either binding long dsRNA to prevent Dicer‐mediated cleavage (e.g. Flockhouse virus B2 protein 4) or binding siRNAs to prevent active‐RISC formation (e.g. p19 protein of tombusviruses 5, 6). From a biotechnology standpoint, p19 and other VSRS offer a unique ‘molecular toolbox' for manipulating and probing protein–RNA interactions in both *in vitro* and living systems; their specialized binding properties and amenability to engineering and multiplexing have made them powerful tools for probing RNA biology (reviewed in Ref. 1, 7). In‐depth understanding of VSRS–RNA interactions and the ability to engineer novel properties is central to these applications.

The p19 protein is the VSRS expressed by tombusviruses, is the most widely studied of the VSRSs. The unique features of the p19 protein are evident from structural and biochemical studies that demonstrate p19's ability to bind to small dsRNAs with size specificity and independently of the nucleotide sequence of the RNA 8, 9. p19 evolved to bind with picomolar affinity to Dicer‐generated, 21‐nt viral‐derived (v)siRNAs, which are 19 base pairs in length of perfectly duplexed Watson–Crick base pairs with 2‐nt 3' overhangs. During viral infection of a host plant, p19 preferentially binds these vsiRNAs, preventing their incorporation into RISC, and does not bind endogenous small RNAs, such as miRNAs 10. When employed recombinantly (in other biological systems or in the absence of viral infection), however, p19 binds other endogenous RNA ligands such as microRNAs (miRNAs), albeit with reduced affinity 10, 11, 12.

## p19 binding to miRNAs

miRNAs are endogenous small RNAs that are potent regulators of gene expression, are critical in host–pathogen interactions and can serve as biomarkers of disease 13. New strategies for detection, quantification and sequestration of miRNAs in living systems and in biological samples such as human serum have been critical for understanding miRNA function and modulating their activity towards human therapeutics. Because of its unique ability to bind small RNA duplexes of any sequence, p19 has been applied in a range of creative strategies for small RNA detection and sequestration 7, 14, 15, 16, 17, 18, 19, 20, 21, 22. miRNA duplexes, before being unwound by RISC, are very similar to p19's canonical ligands, 21‐nt vsiRNAs, except that they are 21–23 nt long and typically contain numerous non‐Watson–Crick base pair mismatches in their sequence 23, 24. These mismatches are predicted to alter p19's ability to bind these RNAs with high affinity 10, 12.

Mismatches and bulges in dsRNA structure are important determinants of intermolecular recognition, as they can cause distortions in the helical backbone which can be specifically recognized by RNA binding proteins 25, 26. Structural investigations of the Argonaute family have illustrated how mismatches can influence specificity of protein–RNA interactions 27, 28, 29, 30. For example, human Argonaute‐2 forms extensive hydrophobic and van der Waals interactions with the minor groove of the miRNA–target complex in the seed region of the miRNA, allowing high‐affinity interactions with a target RNA with perfect complementarity to the miRNA seed region 31. This is in contrast to the p19 binding site, which largely forms electrostatic interactions with the dsRNA backbone. It has been demonstrated that p19 has different propensities to bind perfectly duplexed RNAs and mismatched RNAs both *in vitro* and *in vivo* 10, 11, 12, but the structural basis for how mismatches impact p19's ability to bind small RNA duplexes has not been well understood.

## Engineering p19's binding site to accommodate miRNAs

Base pair mismatches in miRNAs alter p19's ability to bind these RNAs with high affinity 12. The noncanonical structure of miRNAs is not well accommodated by p19, suggesting that p19 has evolved with high selectivity towards canonical siRNA. Since p19 has been applied in biotechnology for miRNA detection and for binding miRNAs *in vivo*, engineering the p19 binding site to allow enhanced affinity for specific patterns in miRNA secondary structure would broaden p19's applicability for miRNA detection and sequestration.

We have previously observed that a single point mutation to p19's binding site at the threonine 111 position to either a histidine (p19‐T111H) or a serine (p19‐T111S) leads to a ~50‐fold increase in the binding affinity of p19 for miR‐122 (Fig.**** 1) 12. Mutations to other positions in the binding site predicted to also increase favourable interactions with miR‐122 (T122, V69 and Y73) did not result in an enhancement of binding affinity 12. Expanded mutagenesis at this site indicated that hydrogen bonding potential at position 111 is important, as mutating the threonine to an alanine (p19‐T111A) resulted in a >5‐fold decrease in affinity for the miR‐122 duplex, compared to wild‐type p19 (p19‐WT). Surprisingly, the serine and the histidine mutations did not alter the protein's ability to bind siRNA, but caused the same large enhancement of p19's binding affinity for miRNA. Considering the substantially different side‐chain structures of serine and histidine, we wondered how both p19 mutants have equivalently potent increases in RNA binding affinity compared to wild‐type. We therefore sought to understand the structural basis of increased affinity of these mutants. Herein, we report the structures of CIRV p19‐WT and the mutants p19‐T111S and p19‐T111H in complex with RNA duplexes determined by X‐ray crystallography. Comparison to previous p19 structures and biochemical studies reveals how mutations at position 111 alter hydrogen bonding in the network of water molecules at the RNA–protein interface. These results indicate an unexpected role for the solvent in mediating RNA–protein recognition and suggest new approaches to further altering the binding properties of p19.

**Figure 1:** Depiction of the relative affinities of wild‐type and mutant p19 proteins towards siRNA and the human miR‐122 ligands. The p19 residues predicted to be interacting with the mismatch regions in the secondary structure of miR‐122 were mutated in order to potentially create new, high‐affinity binding interactions. Substitution of Thr111 with a serine or histidine residue resulted in high‐affinity binding to miR‐122 without altering its affinity for siRNA 12.

## Materials and methods

### Protein expression and purification

Full‐length CIRV p19‐WT, p19‐T111S and p19‐T111H constructs were cloned into the pHis‐parallel 2 vector 32. Constructs of CIRV p19‐WT, p19‐T111S and p19‐T111H, which are codon‐optimized for *E. coli* expression, were amplified from pTriEX vectors (as in Ref. 12) using the following primers (5'‐3′), forward primer: gtcatgccatggaacgcgctatcc and reverse primer: gtcatg ctcgagttactcgctttctttcttgaagg, and ligated into the pHis‐parallel 2 vector using NcoI and XhoI restriction sites. The protein expression construct encodes an N‐terminal 6‐histidine tag followed by a TEV protease cleavage site. All plasmids were confirmed by DNA sequencing.

Plasmids were transformed into BL21 DE3 cells, and cultures were grown from single colonies in 150 mL LB+ 100 mm ampicillin cultures overnight at 37 °C shaking at 220 rpm. The next day, 1‐L flasks were inoculated with starter culture to an OD of 0.1 and grown in LB+Amp at 37 °C until an OD 0.4–0.5. Protein expression was then induced by addition of IPTG (1 mm, final) at 25 °C for 4 h. Cells were harvested by centrifugation, resuspended in lysis buffer (50 mm Tris pH 8.0, 0.3 m NaCl and 0.5 mm TCEP) and lysed by a single pass through a M‐110P homogenizer (Microfluidics, Westwood, MA, USA).

Protein purification was performed by gravity filtration of the bacterial lysate suspended in lysis buffer (50 mm Tris pH 8.0, 0.3 m NaCl and 0.5 mm TCEP) over Nickel resin (HisSelect Nickel Affinity Gel, P6611, Sigma, prepared according to manufacturer's recommendations). The resin was washed with wash buffer (50 mm Tris pH 8.0, 0.3 m NaCl, 60 mm imidazole and 0.5mm TCEP). The his‐tagged p19 was eluted with 50mm Tris pH 8.0, 0.3 m NaCl, 0.3 m imidazole and 0.5mm TCEP and was dialysed in buffer (50 mm Tris (pH 8), 300 mm NaCl and 1 mm TCEP) with 2 mg of tobacco etch virus (TEV) protease at 4 °C overnight to remove the N‐terminal 6‐histidine tag. Gravity filtration over Nickel resin (HiTrap Chelating HP, GE Healthcare, 17‐0408‐01, Lafayette, CO, USA) allowed capture of the portion of the his‐tagged p19 molecules which remained uncleaved, as well as the TEV protease (containing a 6‐histidine tag). The tag‐free p19 protein was then concentrated using Amicon Ultra‐5 Centrifugal Filter tubes (Millipore Sigma UFC801024, Etobicoke, Ontario, Canada) to 0.5 mL and purified by size‐exclusion chromatography on a Superdex 200 10/30 (GE Healthcare Life Sciences) in FPLC buffer [20 mm Tris (7.4), 150 mm NaCl and 1 mm TCEP].

Purities of p19 preparations were assessed by SDS/PAGE and visualization by Coomassie staining. The concentration of purified protein was determined by light absorbance at 280 nm using a Thermo Scientific™ NanoDrop (Montreal, QC, Canada) 2000 spectrophotometer, with the calculated extinction coefficient of 34 950 m ^−1^·cm^−1^ for p19. Protein samples were stored at 4 °C for a maximum of 48 h until application to crystallization trials.

### Oligonucleotides

GL2 siRNA is 21 nucleotides long with two nucleotide overhangs, in which we used modified deoxythymidine nucleotides for the overhangs. The RNA was custom‐ordered from Thermo Scientific and was prepared as follows by the manufacturer: the individual strands were 5′ phosphorylated, converted to the 2′ hydroxyl, annealed and desalted, and purified by polyacrylamide gel electrophoresis. The sense strand (CGUACGCGGAAUACUUCGAUU) and antisense strand (UCGAAGUAUUCCGCGUACGUU) were annealed to allow siRNA duplex formation. We resuspended the purchased annealed siRNA duplex in DEPC‐treated water.

### Crystallization and data collection

Protein–RNA complexes were formed by mixing 1.2 molar equivalents of RNA with 1 molar equivalent of protein (2 mg·mL^−1^) for 1 h at 4 °C. Crystals of p19–RNA complexes were grown using hanging drop vapour diffusion at 4 °C. Drops contained a 1 : 1 ratio of protein–RNA complex (0.8 μL of 2mg·mL^−1^) to 0.8 μL reservoir solution containing 3–12% PEG 1500, 100 mm sodium acetate pH 4.6 and 10–40 mm MgCl_2_. The best crystals were grown from drops that were seeded with smaller crystals, which had been crushed via vortexing with seed beads (Hampton Research, HR2‐320), and streaked through the drops using one of Cupcake the cat's whiskers. The crystals developed a hexagonal morphology over the course of 1–2 weeks at 4 °C. The crystals were harvested with nylon loops, cryo‐protected in the reservoir solution supplemented with 30% ethylene glycol (final), and flash‐frozen in liquid N_2_. Data were collected under cryogenic conditions at beamlines 12‐2 at Stanford Synchrotron Radiation Lightsource (SSRL) 33.

### Structure determination

The p19–siRNA crystals diffracted X‐rays to a maximum resolution of 2.3–1.8 angstroms. The data collected from the p19–siRNA complexes (p19‐WT, p19‐T111S and p19‐T111H) were indexed and scaled using XDS 34 and CCP4 35 into the space group P1. The structure was solved by molecular replacement using PHENIX 36 and a previously determined structure of CIRV p19 in complex with an siRNA duplex as the search model (PDB code: 1RPU) 8. p19:miRNA crystals also diffracted to ~2.5 angstrom, but the crystals displayed diffraction patterns consistent with multiple crystal lattices and could not be assigned to a consistent space group with confidence. We were therefore unable to index and scale diffraction data, and thus were not able to generate a model of p19 in complex with miRNA‐122. Models were built using Coot 37 and submitted to XYZ coordinate, TLS and B‐factor refinement using PHENIX. Model building and refinement were continued iteratively. Water molecules were identified by manual inspection of the electron density maps. All structure figures were generated with PyMOL (Schrödinger, LLC). All of the p19–RNA structures were refined against a common R‐free data set.

## Results and Discussion

### Impact of p19‐T111X mutation on overall architecture of the p19 dimer

In pursuing structural basis for the high affinity of the p19‐T111X mutants towards the mammalian miR‐122, we first sought to understand the impact of the mutations on the overall architecture of the p19 protein. Crystals of wild‐type CIRV p19 (p19‐WT) and the p19 mutants p19‐T111H and p19‐T111S in complex with a perfectly duplexed siRNA were grown and were found to diffract to 2.2 to 2.6 Å (Table 1). These data were then used for detailed analysis of the effects of p19‐T111X mutants.

**Table 1:** Crystallographic data processing and refinement statistics for wild‐type p19 (WT) as well as p19‐T111S and p19‐T111H mutants

p19 crystal	WT	T111S	T111H
PDB ID	6BJV	6BJH	6BJG
Space group	P1	P1	P1
Unit cell dimensions			
a, b, c (Ǻ)	46.6, 49.0, 54.9	45.8, 46.2, 54.2	45.8, 46.2, 54.2
α, β, γ (°)	109.4, 111.1, 96.8	109.9, 122.1, 95.5	109.9, 112.1, 95.5
Molecules per asymmetric unit	2	2	2
Data collection			
Wavelength (Ǻ)	0.9795	0.9795	0.9795
Resolution	46.8–2.2	40.0–2.6	40.0–2.3
Number of reflections	18756	9153	15444
Completeness (%)	93.5 (68.9)	85.3 (72.5)	87.6 (78.2)
Redundancy	2.2	1.9	3.9
*I*/sigma	20.7 (1.84)	5.3 (2.2)	13.3 (6.1)
*R*_merge_	14.7 (74.1)	7.5 (25.1)	5.4(14.5)
*R*_pim_	9.2 (47.8)	7.5 (25.1)	3.1(8.6)
Refinement			
Resolution (Ǻ)	46.8–2.2	34.0–2.6	34.8–2.3
*R*‐free	29.71	27.70	25.57
*R*‐work	26.00	22.37	21.21
RMS deviation *Z*‐scores			
Bond distances (Ǻ)	0.002	0.002	0.002
Bond angles (°)	0.492	0.437	0.455
Number of atoms			
Nonhydrogen, protein	5813	5770	5799
Nonhydrogen, RNA	4437	4375	4377
Water	65	129	121
Ramachandran plot			
Total analysed			
Preferred (%)	92.76	91.40	96.44
Allowed (%)	6.55	8.24	3.56
Outliers (%)	0.69	0.36	0

*R*_merge_ = ∑_*h*_∑_*i*_|*I*_*h*_−*I*_*hi*_|/∑_*h*_∑_*i*_ *I*_hi_, where *I*_*h*_ is the mean of *I*_hi_ observations of reflection *h*. Numbers in parentheses represent data for the highest resolution shell.

*R*_work_ and *R*_free_ = ∑||*F*_obs_|−|*F*_calc_||/∑|*F*_obs_| × 100 for 95% of the recorded data (*R*_work_) or 5% of the data (*R*_free_).

The p19 structures reported here are in agreement with the previously published structure of CIRV p19 with the same characteristic features and binding site interactions observed 8. The p19 protein associates as a tail‐to‐tail homodimer, forming a concave 8‐stranded beta‐sheet binding surface, which engages the sugar‐phosphate backbone of the bound siRNA through electrostatic and hydrogen bond interactions. The protein does not make contact with the nitrogenous bases of the RNA along the length of the duplex, allowing p19 to bind small RNA duplexes independently of RNA sequence. We also observed the characteristic ‘molecular calliper' nature of the p19 dimer, where tryptophans W39 and W42 provide stacking interactions on the 19th base pair of the RNA duplex. These stacking interactions provide stabilizing energy between the protein and the RNA duplex 19 base pairs in length, contributing to p19's high affinity for siRNA ligands and garnering size specificity to p19's interactions 8, 38. p19's affinity drops dramatically for binding RNA duplexes shorter or longer than 19 base pairs 8, 11, 12.

Next, we examined the structures of the p19‐T111X mutants to assess the impacts of the amino acid substitution on the overall topography of the p19 dimer. As displayed in Fig.**** 2 **,** the p19‐T111H and p19‐T111S structures align very consistently with the p19‐WT structure. In Fig. 2A, we show that the p19‐T111H dimer overlaps with WT with an overall RMSD of 0.315 angstroms, and in Fig. 2B**,** we show that p19‐T111S overlaps with WT with an overall RMSD of 0.471 angstroms. This result is in agreement with previously published circular dichroism and thermal melt analysis, which suggested that the p19‐T111H and p19‐T111S mutations did not significantly alter the secondary structure of the protein 12. The consistency of the p19‐T111H and p19‐T111S structures with WT is further to be expected given that the mutants' affinity for siRNA was not altered from WT (*K*_d_ = 0.2 nm) 12. The structures therefore support biochemical evidence, indicating that the p19 binding site is amenable to mutation at the 111 site without impacting the architecture of the protein dimer. The structural alignments suggest that p19‐T111X mutants largely retain their p19‐WT secondary structure and imply a similar binding mode with different RNA ligands.

**Figure 2:** Alignments of p19 mutants with wild‐type p19 (A) Alignment of p19‐WT (grey) with T111H mutant (green), rotated 180 degrees in right‐hand panel. Aligning the p19 dimers resulted in an overall RMSD of 0.315 angstroms, indicating that the T111H mutant does not have substantial impact on the architecture of the p19 dimer and the siRNA binding site. (B) Alignment of p19‐WT (grey) with T111S mutant (yellow), rotated 180 degrees in right‐hand panel. Aligning the p19 dimers resulted in an overall RMSD of 0.471 angstroms, indicating that the T111S mutant does not have substantial impact on the architecture of the p19 dimer and the siRNA binding site.

### p19‐T111X mutants

In pursuing structural determination of the p19 mutants, we sought to examine specific interactions between the protein and the miRNA which could explain the observed 50‐fold enhancement from WT on miR‐122 binding affinity, without altering the protein's affinity for siRNA ligands 12. The change in binding affinity we have observed is associated with an approximate free energy change between p19‐WT and p19‐T111H/S mutants (ΔΔG) of 2.3 kcal·mol^−1^. This change in the free energy upon binding could be due to the T111H or T111S mutation providing a favourable change in enthalpy (ΔH), through generating increased contacts between the binding site and the miRNA (e.g. ~2 hydrogen bonds). These could be direct interactions with the secondary structure of the miRNA or could be an increase in the number of water‐mediated hydrogen bonds that are prevalent in the p19–RNA binding site. Therefore, the orientation and organization of hydrogen bonds associated with the mutated residues are expected to play a key role in providing the free energy difference associated with binding.

The p19 mutants p19‐T111S and p19‐T111H contain two chemically distinct mutations that give rise to nearly identical changes in the RNA binding properties of p19 12. Initial efforts to understand the structural basis for this observation focused on determining structures of these mutants p19 in complex with miR‐122. Although p19‐miR‐122 crystals could be grown, diffraction patterns indicated the presence of multiple crystal lattices and no space group could be assigned (see Materials and methods). We therefore focused our efforts on determining structures of p19‐T111H/T111S mutants bound to canonical siRNA ligands.

The p19‐T111 site of each p19 monomer is positioned on the second beta‐strand (counting the beta‐strands from N‐C termini) and the two T111 sites in the dimer insert into the minor groove of the central region of the bound RNA, in proximity to the RNA backbone (Fig.**** 3). Figure 3A displays the structure of p19‐T111H in complex with siRNA, with the central base pair of the RNA duplex highlighted in blue. We observe in the H111 model that the protein engages an ordered water molecule and forms a hydrogen bond with the bridging oxygen on the siRNA backbone (Fig. 3B). The position of this contact is with the central A10‐U10' base pair of the siRNA. Importantly, this is where we expect the central C:A mismatch of the miR‐122 molecule to cause alterations in the duplex structure and the hydrogen bond network that account for the ΔΔG of binding. For comparison, Fig. 3C displays a structure determined separately (PDB code: 4JK0), where a glutamine mutation has been introduced at the same 111 site in the p19 protein from the tobacco bushy stunt virus (TBSV). p19 is highly conserved among tombusviruses, and the TBSV p19 and the CIRV p19 share 86% amino acid identity and the same protein architecture 8, 9. This p19‐T111Q mutant displays novel hydrogen bonds with the 2′ OH of the backbone at the central base pair, as well as with the amino group of the nucleotide base (guanine 9). These structures show how mutants at position‐111 with longer side chains can reach into the minor groove and contact the nucleotide bases. In Fig. 3D, the p19‐T111S structure does not show direct or water‐mediated contacts with the siRNA, showing no discernable differences in the interactions observed compared to the p19‐WT structure at that site (Fig. 3E). Each mutation at the T111 site, therefore, displays a different mode of interaction with its bound RNA, where additional opportunities for water‐mediated hydrogen bonds exist in T111H and T111Q. Given that the chemical differences between T111S and WT involve the placement of a single methyl group, it is logical to conclude that the T111S mutant contains greater flexibility to engage the miR‐122 ligand. Thus, flexibility of direct and water‐mediated interactions is likely what allows chemically distinct mutants to stabilize a variety of RNA ligands.

**Figure 3:** Structural analysis of p19‐T111X mutants. (A) Crystal structure of p19 mutant histidine‐111 (‘H111') in complex with siRNA. p19 monomers in yellow and green, with H111 residues highlighted in red, and the central base pair highlighted in blue. (B) The H111 residue engages an ordered water molecule for a hydrogen bond (dashed lines) with the bridging oxygen on the siRNA backbone (adenine 10). (C) The Q111 residue makes novel hydrogen bonds with the 2′ OH of the backbone at the central base pair, as well as with the amino group of the nucleotide base (guanine 9) (PDB code: 4JKO). (D) The serine‐111 (‘S111') residue does not display any direct contacts with the siRNA backbone, with no discernable change in the interactions observed compared to the wild‐type threonine‐111 (T111) structure (E).

### Water‐mediated hydrogen bond network in binding site

Water molecules in protein–RNA binding sites contribute to binding affinity, providing hydrogen bond opportunities between the protein binding site and RNA, as well as shielding of unfavourable charge interactions between the two molecules 39, 40, 41. Further, water can contribute to specificity of ligand interactions, as observed for the tet repressor complex 42 and Ago2–target interactions 43. In the p19 structures reported here, we observe a network of waters in the binding site that appears to aid in making contacts between the protein and the minor groove of the bound RNA. The presence of a water network in the p19 binding site provides several extra hydrogen bonding opportunities that may contribute to the favourable enthalpic binding energy between p19 and its bound RNA. A similar idea was proposed for the involvement of a water‐mediated hydrogen bond network in the binding site of TBSV p19 9.

In comparing the water molecules in the binding site between the p19‐WT and the p19‐T111H mutant, we observe that most of the water molecules shift positions in the binding site. In examining the hydration near the 111 site, we observe that an ordered water molecule engaged by the WT threonine is displaced by the histidine in the p19‐T111H structure (Fig. 4). This observation serves as an example of how water‐mediated contacts may shift with mutation to binding site residues and indirectly impact interactions with the bound RNA. The central mismatch in miR‐122 would likely alter the water‐mediated hydrogen bond network in the binding site, as has been observed with structural comparison of perfectly duplexed to mismatched RNAs 44, 45. These observations suggest that T111X mutations can shift the binding affinity towards different RNA ligands through a shift in the water‐mediated hydrogen bond network in the binding site.

**Figure 4:** Examining water‐mediated interactions between p19 and bound RNA at position 111. Three‐way alignment of p19‐WT (grey) p19‐T111H (green) and p19‐T111S (yellow) structures reveals that an ordered water molecule engaged by both the WT threonine (grey) and the mutant serine (yellow) through a hydrogen bond is displaced by the histidine in the p19‐T111H structure (green).

The structures determined here highlight T111 as uniquely positioned for access to the nucleotide bases along the central base pair of the bound RNA duplex, which is the position of the central mismatch of miR‐122. In support of this argument, others have observed in structures of p19 in complex with CNG repeat RNAs containing G:U and U:U mismatches, another form of noncanonical RNA duplex, that p19 is able to influence the geometry of the RNA helix, stabilizing irregular dsRNA geometries into more regular Watson–Crick formations (PDB 4KTG, 4J5V, 4KNQ, 4JNX, 4JGN, 4KQO and 4J39) 44, 45. This is consistent with an induced fit model for binding of the RNA ligand and supports the notion that p19 largely retains its structure in complex with noncanonical RNA ligands. Given the unique position of the 111 residue in relation to the central mismatch of miR‐122, our data suggest that H111 and S111 are able to enhance p19's affinity for miR‐122 by stabilizing the central mismatch of the miRNA more effectively than T111, either through direct or water‐mediated hydrogen bonding which would support a more favourable helical geometry of the RNA duplex.

The structures presented here offer insight into the rearrangement of hydrogen bonding and ordered waters between the WT and mutant p19 proteins in the protein–RNA binding site, suggesting that these may be responsible for alterations in the Δ*H* of RNA binding. The alterations in ordered water molecules observed in these structures lend insight into how mutations to the binding site can engage water molecules to provide novel stabilizing interactions with their RNA ligands, which could contribute favourable enthalpic contributions to the increase in affinity for mismatched RNA ligands associated with T111H and T111S mutations.

## Conclusions

The p19 protein is a unique platform for studying small RNA duplexes, and engineering its properties will further broaden its applications in small RNA detection and sequestration. We report here that mutations at the T111 site do not alter the overall architecture of the p19 dimer but instead are associated with subtle changes in direct and water‐mediated hydrogen bond networks with its RNA ligand. It is the unique position of the T111 residue along the central axis of the RNA duplex which positions it to provide stabilizing interactions with the central mismatch of the miRNA duplex of miR‐122, thereby allowing a higher affinity interaction. This is supported by comparing these structures with previously reported structures of p19 with mismatched RNAs, which show that p19 stabilizes the structure of mismatched RNA duplexes to form a more regular Watson–Crick backbone geometry. The X‐ray crystal structures of CIRV p19 and mutants p19‐T111S and p19‐T111H in complex with siRNA reported here will aid future structure‐based rational design of p19 mutants for binding noncanonical RNA molecules, such as miRNAs. Future work will aim to resolve the relative enthalpic and entropic contributions of p19–RNA interactions, and the impact of mutation on the thermodynamic landscape of p19–RNA interactions. In understanding the specific interactions guiding high‐affinity interactions with miRNA mismatches, we envision a system that we can rationally engineer for targeting specific small duplex RNA ligands in biological systems, as was recently done with the RNA Recognition Motif (RRM) for influencing miR‐21 activity 46. Furthermore, these approaches for rationally engineering ligand specificities can be combined with other p19‐based technologies, such as p19 with incorporated unnatural amino acids which allows visualization of small RNA capture and delivery in living systems 47.

## Conflict of Interest

The authors declare no conflict of interest.

## Author contributions

DF, IM and JP designed and conceived of the project. DF and NS collected the data. DF, JP and IM interpreted the results. DF wrote the manuscript with conceptual and editing help from JP and IM.
